RETRACTED

# Clinical Study on the Differential Diagnosis of High Myopia Astigmatism and Subclinical Keratoconus in Adolescents by Pentacam Anterior Segment Analyzer

**DOI:** 10.1155/2022/6370791

**Published:** 2022-05-16

**Authors:** Yimeng Ruan, Ying Zhang, Xiaohong Ying

**Affiliations:** ^1^Department of Ophthalmology, Ningbo First Hospital, No. 59, Liuting Street, Ningbo 315010, Zhejiang, China; ^2^Department of Ophthalmology, Xiaoshan Hospital Affiliated to Hangzhou Normal University, No. 728, Yucai North Road, Xiaoshan District, Hangzhou 311002, Zhejiang, China

## Abstract

To explore the clinical value of Pentacam anterior segment analyzer in differential diagnosis of high myopia astigmatism and subclinical keratoconus in adolescents. The study included 100 teenagers with ophthalmic diseases treated at our hospital between July 2015 and August 2021, including 58 individuals with simple high myopia astigmatism (73 eyes in the simple high myopia astigmatism group) and 42 teenagers with subclinical keratoconus (51 eyes in the subclinical keratoconus group). The corneal parameters of the two groups were measured with a Pentacam anterior segment analyzer, and we compared the thinnest corneal thickness, anterior (posterior) vertex height of the thinnest point of the cornea, index of vertical asymmetry (IVA), index of height descent (IHD), and the average corneal pachymetric progression index. The receiver operating characteristic curve (ROC) was drawn to evaluate the value of various parameters and combined diagnostic factor Y in the differential diagnosis of high myopia astigmatism and subclinical keratoconus. The thinnest region of the cornea in the subclinical keratoconus group was less than that in the simple high myopia astigmatism group, while the anterior (posterior) vertex height of the thinnest point of the cornea, index of vertical asymmetry (IVA), index of height decentration (IHD), and average corneal pachymetric progression index were higher than those in the simple high myopia astigmatism group (*P* < 0.05). For the differential diagnosis of high myopia astigmatism and subclinical keratoconus, the combined diagnostic factor Y, anterior (posterior) vertex height, IVA, IHD, and mean corneal progression index were 0.808, 0.833, 0.868, 0.847, 0.684, and 0.926 (*P* < 0.05). The AUC of the combined diagnostic factory was the largest, which was significantly different from that of the anterior vertex height of the thinnest point of the cornea (*Z* = 3.280), the posterior vertex height of the thinnest point of the cornea (*Z* = 3.205), IVA (*Z* = 2.764), IHD (*Z* = 2.237), and the average corneal progression index (*Z* = 4.125) (*P* < 0.05). Using the Pentacam anterior segment analyzer, differential diagnoses can be made for high myopia, astigmatism, and subclinical keratoconus.

RETRACTED

## 1. Introduction

Keratoconus is a primary noninflammatory corneal disease characterized by conus-like protrusions of the cornea, which can cause vision loss, irregular myopia, and astigmatism and bring great adverse effects on patients' daily life, work, and study [1, 2]. The latest research results show that the prevalence and incidence of keratoconus are estimated to be 0.2 to 4790 per 100000 and 1.5 to 25 per 100000 per year, respectively. The high prevalence and incidence of keratoconus usually occur in people between 20 and 30 years old. The differences were attributed to geographical location and race, definition and diagnostic criteria of keratoconus, study design, and differences in age and cohort of subjects evaluated. It is clinically believed that patients with keratoconus have no specific early signs and symptoms, similar to those with high myopia, astigmatism, and amblyopia. However, they all show decreased vision, which is also the main reason for the misdiagnosis of subclinical keratoconus [3]. With the rapid development of medical technology, the Pentacam anterior segment analyzer has been widely used in diagnosing ophthalmic diseases. Compared with traditional corneal topography, the Pentacam anterior segment analyzer is more accurate and repeatable and can accurately obtain the corneal surface height, providing reliable diagnostic information for clinical treatment [4, 5]. Researchers have also noted [6] that the Pentacam anterior segment analyzer can distinguish between simple high myopia astigmatism and subclinical keratoconus by reflecting subtle differences in corneal morphology. By the way, clinically, we often adopt the “diagnostic factor Y” to intuitively react to the dynamic, changing process of the cornea, and the situation of altered corneal biomechanics. To this end, this study retrospectively analyzed the clinical data of 100 patients with ophthalmic diseases treated in the Ophthalmology Department of Ningbo First Hospital from July 2015 to August 2021 and explored the clinical value of Pentacam anterior segment analyzer in the differential diagnosis of simple high myopia astigmatism and subclinical keratoconus.

## 2. Materials and Methods

### 2.1. General Information

During the study period of July 2015 to August 2021, 100 teenage patients with ophthalmic diseases were evaluated, including 58 patients with simple high myopia astigmatism (73 eyes, simple high myopia group) and 42 patients with subclinical keratoconus (51 eyes, subclinical keratoconus group). There were 31 boys (39 eyes) and 27 girls (33 eyes) in the simple high myopia astigmatism group; the age ranged from 16 to 18 years, with an average age of (16.96 ± 2.05) years. In the subclinical keratoconus group, there were 26 boys (30 eyes) and 16 girls (21 eyes); the age ranged from 16 to 18 years, with an average age of (16.87 ± 2.11) years. A comparison of baseline data such as gender ratios and age distributions of the two groups was performed using the SPSS 21.0 statistical software. No significant difference between these data were observed (*P* > 0.05).

RETRACTED

### 2.2. Selection Criteria

#### 2.2.1. Inclusion Criteria

Simple high myopia astigmatism group: (1) Age range: 16–18 years old; (2) Astigmatism ≥2.5 D, corrected visual acuity ≥0.8; (3) No contact lens use within 1 month of examination; (4) Complete clinical data; (5) No family history of keratoconus; (6) No family history of hereditary eye disease. The subclinical keratoconus group: (1) Age range: 16–18 years old; (2) Astigmatism ≥2.5 D, corrected visual acuity ≥0.8; (3) Slit-lamp microscope showed no change in corneal morphology; (4) The corneal topography met the Rabinowitz diagnostic criteria [7]; (5) Complete clinical data; (6) No family history of hereditary eye diseases.

#### 2.2.2. Exclusion Criteria

(1) Patients with chronic inflammation of the ocular surface, uveitis, and other ocular diseases; (2) Those with a history of ocular trauma or eye surgery; (3) Those with systemic diseases.

### 2.3. Inspection Method

All patients underwent routine visual inspection as well as examination by slit-lamp microscopy. Detection of corneal parameters with Pentacam anterior segment analyzer: the examination methods and precautions were clearly explained to patients and their families and the patients were assisted in maintaining a comfortable sitting position. The instrument did not directly touch the eye's surface during the examination. After turning on the device, the patient's name, age, gender, and other clinical information was entered and the patient was instructed patient to place their chin on the jaw rest, the forehead close to the forehead band, and to open both eyes and stare at the circle in the blue light ahead. The inspection technician moved the joystick for manual focus. The device completed the scan of the anterior segment structure within 2 seconds, obtained high-definition images, recorded the thinnest corneal thickness, the anterior (posterior) vertex height of the thinnest point of the cornea, index of vertical asymmetry (IVA), index of height decentration (IHD), and mean corneal progression index. Each eye was measured 3 times, and the average value of each parameter was entered into the database.

RETRACTED

### 2.4. Data Processing

SPSS 21.0 was used for data processing, and Kolmogorov–Smirnov normality test analysis showed that the corneal parameters of the two groups of patients were all in a normal distribution, expressed as ($\bar{x}$ ± *s*), and an independent *t*-test was performed for comparison between groups. The indexes were imported into the logistic regression model, the regression equation was constructed, the joint diagnostic factor Y of each parameter index was obtained, and each parameter index and the joint diagnostic factor Y were entered into the MedCalc software. Next, the receiver operating characteristic curve (ROC) was drawn, and the area under the curve (AUC) was compared. The differential diagnosis value of each parameter index was compared, and the combined diagnostic factor Y for simple high myopia astigmatism and subclinical keratoconus. *P* < 0.05 was considered to be statistically significant.

## 3. Results

### 3.1. Comparison of the Parameters of the Two Groups

The thinnest corneal thickness in the subclinical keratoconus group was smaller than that in the high myopia astigmatism group. In contrast, the anterior vertex height of the thinnest point of the cornea, the posterior vertex height of the thinnest point of the cornea, IVA, IHD, and average corneal pachymetric progression index (PPI) were significantly higher than those in the high myopia astigmatism group (*P* < 0.05), as shown in Table 1.

### 3.2. Regression Equation of Joint Diagnostic Factor *Y*

According to the logistic regression analysis results in Table 2, the regression equation of the joint diagnostic factor Y was established:

(1) $$\begin{array}{c} Y=\frac{e^{0.206X_{1}+0.536X_{2}+0.661X_{3}+0.713X_{4}+0.549X_{5}+0.436X_{6}-13.581}}{1+e^{0.206X_{1}+0.536X_{2}+0.661X_{3}+0.713X_{4}+0.549X_{5}+0.436X_{6}-13.581}}. \end{array}$$

Among them, *X*_1_-*X*_6_ represent the thickness of the thinnest cornea, the anterior vertex height of the thinnest point of the cornea, the posterior vertex height of the thinnest point of the cornea, the detection data of IVA, IHD, and the average corneal pachymetric progression index.

### 3.3. Analysis of the Differential Diagnosis Value of Various Parameters for High Myopia Astigmatism and Subclinical Keratoconus

ROC curve analysis showed that the AUC of the anterior vertex height of the thinnest point of the cornea, the posterior vertex height of the thinnest point of the cornea, the detection data of IVA, IHD, the average corneal pachymetric progression index and the joint diagnostic factor Y were 0.808, 0.833, 0.868, 0.847, 0.684, and 0.926 and were significantly higher than those in the high myopia astigmatism group (*P* < 0.05). Medcale analysis showed that the AUC of joint diagnostic factor Y was the largest, and there were statistically significant differences between AUC and anterior vertex height of the thinnest point of the cornea (*Z* = 3.280), posterior vertex height of the thinnest point of the cornea (*Z* = 3.205), IVA (*Z* = 2.764), IHD (*Z* = 2.237), and average corneal pachymetric progression index (*Z* = 4.125) (*P* < 0.05). Compared with high myopia astigmatism group (*P* < 0.05), as shown in Table 3 and Figure 1.

RETRACTED

## 4. Discussion

It has been reported that corneal refractive power accounts for more than 70% of the total refraction of the eyeball and is the most important refractive surface of the human body [8]. Therefore, corneal refractive surgery is one of the most effective methods to treat keratoconus, which helps to improve the vision of patients and achieve the therapeutic goal of correcting refractive errors. In the early stages of keratoconus, symptoms can mimic myopia and astigmatism, making early detection difficult. It is easy to miss the most optimal time for treatment [9]. Therefore, it is of great clinical significance to adopt a scientific and effective diagnostic method for early keratoconus screening.

The anterior cone protrusion of the cornea is the most prominent clinical feature of keratoconus; however, patients with subclinical keratoconus presenting with irregular astigmatism or amblyopia do not have such specific symptoms, complicating the differential diagnosis. The detection of corneal parameters is an effective method for early clinical diagnosis of keratoconus [10, 11]. In recent years, with the broad application of the Pentacam anterior segment analyzer, ideal clinical results have been achieved in the accurate measurement of complex corneas, corneal limbus, and thin corneas [12]. Some studies have pointed out [13] that the use of Pentacam anterior segment analyzer to detect corneal morphological changes can provide accurate data reference for clinical diagnosis of myopia and keratoconus and help guide clinical treatment. Pentacam anterior segment analyzer is a new type of multifunctional ophthalmic instrument, which can achieve 25 scans in 1 s, obtain 25,000 actual elevation points after reflection from the cornea, iris, lens, etc., and finally obtain three-dimensional color images and data [14]. In addition, compared with the previous traditional corneal topography detector, the Pentacam anterior segment analyzer can realize 3D modeling and calculate the thickness of all corneal sites with higher accuracy and repeatability [15].

In this study, we used the Pentacam anterior segment analyzer to measure the corneal parameters of patients with myopia, astigmatism, and subclinical keratoconus. Our results showed that the thinnest corneal thickness in the subclinical keratoconus group was smaller than that in the high myopia flash group. The anterior and posterior vertex height of the thinnest point of the cornea, IVA, IHD, and average corneal progression index were significantly elevated compared to those in the high myopia astigmatism group (*P* < 0.05). Thus, patients with high myopia astigmatism and subclinical keratoconus have significantly different corneal parameters, which is consistent with Hu et al. findings [16]. Muftuoglu et al. [17] also found that the IVA, IHD, and anterior (posterior) vertex height of the thinnest point of the cornea in patients with subclinical keratoconus were higher than those in patients with simple high myopia astigmatism. The above results indicate that utilizing the Pentacam anterior segment analyzer to detect corneal parameter changes can be used as a reference for the differential diagnosis of high myopia astigmatism and subclinical keratoconus. However, for different stages of keratoconus, especially the biomechanical characteristics of suspicious or preclinical keratoconus, we need to further study.

RETRACTED

In addition, this study drew the ROC curve of each parameter index in the differential diagnosis of high myopic astigmatism and subclinical keratoconus. The AUC of the anterior vertex height of the thinnest point of the cornea, the posterior vertex height of the thinnest point of the cornea, IVA, IHD, average corneal progression index, and combined diagnostic factor Y were 0.808, 0.833, 0.868, 0.847, 0.684, and 0.926, respectively. The analysis results revealed that IVA and IHD had the highest AUC among the single index, which indicates that these indexes are the most useful in the differential diagnosis of high myopia astigmatism and subclinical keratoconus. Reasons for this may be that IVA and IHD are important parameters that reflect the symmetry and regularity of the cornea, keratoconus is characterized by lordosis of the cornea, the uneven redistribution of corneal curvature, and IVA and IHD change significantly. Meanwhile, high myopia astigmatism is generally symmetrical, with little change in IVA and IHD according to the Pentacam anterior segment analyzer. Wu et al. [18] selected 32 patients with ophthalmic diseases, used the Pentacam anterior segment analyzer to detect the corneal parameters, and plotted the parameters for the differential diagnosis of high myopia astigmatism and subclinical keratoconus. The ROC curve of the cornea showed that the anterior vertex height of the thinnest point of the cornea, the posterior vertex height of the thinnest point of the cornea, IVA, IHD, average corneal progression index, and combined diagnostic factor Y were 0.816, 0.822, 0.736, 0.773, and 0.922 (*P* < 0.05), which were similar to our study. Analysis of the AUC of each index showed that the AUC of the combined diagnostic factor Y was significantly greater than those of any single index (*P* < 0.05). This finding indicates that the diagnostic accuracy of high myopia astigmatism and subclinical keratoconus can be enhanced by considering the anterior vertex height of the thinnest point of the cornea, the posterior vertex height of the thinnest point of the cornea, IVA, and IHD. In conclusion, there are significant differences in corneal parameters between patients with high myopic astigmatism and subclinical keratoconus. Therefore, the Pentacam anterior segment analyzer can be used to differentiate between high myopia astigmatism and subclinical keratoconus.

RETRACTED

## Figures and Tables

**Figure 1:** ROC curve of various parameters in the differential diagnosis of high myopia astigmatism and subclinical keratoconus.

**Table 1:** Comparison of the parameters of the two groups ($\bar{i}$ ± *s*).

Group	*n*	The thinnest corneal thickness (*μ*m)	The anterior vertex height of the thinnest point of the cornea (*μ*m)	The posterior vertex height of the thinnest point of the cornea (*μ*m)	IVA	IHD	Pachymetric progression index (PPI)
Simple high myopia astigmatism group	73	529.74 ± 57.12	4.37 ± 2.01	8.56 ± 2.74	0.151 ± 0.026	0.010 ± 0.002	1.07 ± 0.23
Subclinical keratoconus group	51	501.35 ± 44.89	6.61 ± 2.34	14.05 ± 3.26	0.248 ± 0.041	0.019 ± 0.006	1.27 ± 0.31
*t*		2.966	5.705	10.149	16.115	11.921	4.124
*P* value		0.004	0.001	0.001	0.001	0.001	0.001

**Table 2:** Logistic regression analysis of each parameter index.

Parameter	Index	OR	95% CI	*P* value
Thinnest corneal thickness	0.206	1.535	1.032∼2.459	0.019
The anterior vertex height of the thinnest point of the cornea	0.536	2.774	1.598∼4.121	0.007
The posterior vertex height of the thinnest point of the cornea	0.661	2.654	1.435∼3.864	0.001
IVA	0.713	3.851	2.106∼7.364	0.001
IHD	0.549	2.714	1.532∼3.976	0.009
The average corneal pachymetric progression index	0.436	2.036	1.299∼3.635	0.011
Constant	−13.581	0.001	—	0.001

**Table 3:** Analysis of the differential diagnosis value of various parameters for high myopia astigmatism and subclinical keratoconus.

Parameter	AUC	95% CI	*P* value	Best cutoff value	Sensitivity (%)	Specificity (%)
Thickness of the thinnest cornea	0.563^*∗*^	0.451∼0.674	0.275	512.35	43.56	32.35
Anterior vertex height of the thinnest point of the cornea	0.808^*∗*^	0.722∼0.893	0.001	5.54	73.58	74.56
Posterior vertex height of the thinnest point of the cornea	0.833^*∗*^	0.755∼0.912	0.001	10.57	75.16	70.37
IVA	0.868^*∗*^	0.796∼0.940	0.001	0.216	79.56	81.35
IHD	0.847^*∗*^	0.767∼0.926	0.001	0.015	78.44	75.23
Average corneal pachymetric progression index	0.684^*∗*^	0.578∼0.790	0.001	1.20	60.35	57.46
Joint diagnostic factor Y	0.926	0.863∼0.989	0.001	0.495	86.94	89.63

RETRACTED

## Data Availability

The simulation experiment data used to support the findings of this study are available from the corresponding author upon request.
